This article has been retracted.

# Genomic Instability in Liver Cells Caused by an LPS-Induced Bystander-Like Effect

**DOI:** 10.1371/journal.pone.0067342

**Published:** 2013-07-09

**Authors:** Igor Kovalchuk, Paul Walz, James Thomas, Olga Kovalchuk

**Affiliations:** Department of Biological Sciences, University of Lethbridge, Lethbridge, Canada; Florida International University, United States of America

## Abstract

Bacterial infection has been linked to carcinogenesis, however, there is lack of knowledge of molecular mechanisms that associate infection with the development of cancer. We analyzed possible effects of the consumption of heat-killed *E. coli* O157:H7 cells or its cellular components, DNA, RNA, protein or lipopolysaccharides (LPS) on gene expression in naïve liver cells. Four week old mice were provided water supplemented with whole heat-killed bacteria or bacterial components for a two week period. One group of animals was sacrificed immediately, whereas another group was allowed to consume uncontaminated tap water for an additional two weeks, and liver samples were collected, post mortem. Liver cells responded to exposure of whole heat-killed bacteria and LPS with alteration in *γ*H2AX levels and levels of proteins involved in proliferation, DNA methylation (MeCP2, DNMT1, DNMT3A and 3B) or DNA repair (APE1 and KU70) as well as with changes in the expression of genes involved in stress response, cell cycle control and bile acid biosynthesis. Other bacterial components analysed in this study did not lead to any significant changes in the tested molecular parameters. This study suggests that lipopolysaccharides are a major component of Gram-negative bacteria that induce molecular changes within naïve cells of the host.

## Introduction

There is clear evidence linking environmental exposures to the onset of carcinomas [1]. Viral infections such as HIV, HCV and HBV have a prominent effect on the development of carcinomas during and after infection. The influence of some bacteria on the effects of genome stability is significant but not widely accepted. *Helicobacter pylori* and its association with the development of gastric cancer is one of the best examples [2]. Presence of a common intestinal bacteria such as *E. coli* may facilitate the development of various malignancies [3].

Bacteria can promote carcinogenesis by induction of chronic infection, leading to disruption of the cell cycle and alterations in cell growth and DNA damage [4]. The association of chronic inflammation with a variety of epithelial malignant tumors has been recognized for many years. For example, squamous carcinoma may develop along the draining sinus in chronic osteomyelitis, and development of adenocarcinoma is a significant risk in patients with chronic inflammatory bowel disease [5]. Even though a link between cancer induction and bacterial infection exists, it is unclear if living or heat-killed cells, or even remnants of the bacteria can trigger genome instability and cancer. Yamamoto *et al*. (1992) conducted tests which exposed urinary bladders to heat killed *E. coli*, which resulted in a 40× enhancement of tumourigenesis in pre-initiated tumour sites [6].

Exposure to bacterial pathogens and/or their components most frequently occurs through consumption of contaminated food or water. Contamination is more frequently identified in rural communities with a high frequency of large livestock farms [7]. Boiling of contaminated water is intended to kill the bacteria and prevent infections, but bacterial remnants such as proteins and LPS may remain intact and have the capability to interact with cells of the gastro-intestinal tract. For example, the liver is exposed to bacterial determinants and/or toxins through its physiological role of detoxification of the blood; specifically, the hepatocytes are involved in clearance of endotoxins [8].

Even though, epidemiological evidence identifies links between bacterial infection and cancer induction, it is still unclear, which/if any, component of the heat-killed bacteria could produce a genomic instability response in naïve cells of the host. Based on the literature, it can be hypothesized that exposure to heat-killed bacteria or their components, causes genomic instability in cells that does not require direct contact with a bacterial cell or its constituents.

Research conducted within recent years has identified that heat- killed bacteria (whether pathogenic *E. coli* O157:H7 or non-pathogenic DH5α) induce genome instability [9]. It was identified that water containing only heat-killed bacteria continued to have the capacity to induce genome instability in the host. The effect remained even after water contaminated with heat-killed bacteria was filtered through a 0.45 µm filter. This indicated that whole bacteria were not required to induce genetic and possibly epigenetic changes, but rather only a single component of the bacteria.

DNA damage is sensed through several independent proteins and protein complexes, depending on the type of damage. Single- and double-strand breaks (SSB and DSB) in the DNA are sensed by three members of the phosphoinositide-3-kinase-related protein kinase (PIKK) family, namely ataxia-telangiectasia mutated (ATM), ataxia-telangiectasia and Rad3-related (ATR) and DNA-dependent protein kinase catalytic subunit (DNA-PKcs) [10]. These checkpoint kinases phosphorylate histone variant H2AX at a serine 139, forming a γH2AX - a sensitive indicator of both DNA damage and DNA replication stress. Double strand breaks are then repaired by either non-homologous or homologous recombination pathways, represented by KU70/KU80 or RAD51/RAD54 protein groups. Another type of common DNA damage is the oxidation and alkylation of nucleotides, and apurinic/apyrimidinic endonuclease 1 (APE1) is the main abasic endonuclease involved in the base excision repair (BER) pathway in mammals [11].

Disruption of a cell cycle caused by bacteria may also lead to increased cell proliferation. One of the proteins, proliferating cell nuclear antigen or PCNA, forms a homotrimer clamp around DNA and acts as a processivity factor for DNA polymerase δ [12]. PCNA is also involved in post-replication repair as well as is able to recruit maintenance DNA methyltransferase 1, DNMT1 to hemimethylated DNA [13]. Thus the analysis of levels of PCNA may serve as a good indication of the activity of DNA replication and DNA repair.

Although little is known about the effect the pathogen infection may have on the chromatin structure of the host, it can be hypothesized that bacterial infection may alter the DNA methylation and chromatin structure of the infected host cells. DNA methylation in animals occurs primarily via the action of *de novo* DNA methyltransferases DNMT3A and DNMT3B and maintenance methyltransferase DNMT1. Whereas hypomethylated DNA is mostly associated with higher gene expression, hypermethylated DNA is typically associated with lower gene expression activity and proteins like MeCP2 bind methylated DNA and recruit histone-modifying proteins and non-histone proteins that reinforce condensed chromatin structure [14].

The purpose of this study was to analyze the level of proteins involved in DNA damage recognition, DNA repair and DNA methylation in liver of animals that consumed heat-killed bacteria and its components DNA, RNA, protein or LPS. We analyzed immediate and delayed effects of consumption of heat killed bacteria and bacterial components and found multiple changes in the expression of aforementioned proteins in response to whole bacteria or LPS but not other components.

## Materials and Methods

### Animal model

Four-week-old C57BL/6 male mice and all subjects were handled and cared for according to the requirements set by the Canadian Council for Animal Care and Use. The procedures have been approved by the University of Lethbridge Animal Welfare Committee. The mice were housed in cages in a virus-free facility with a 12 h light/dark cycle and provided water (with or without treatment) and food pellets *ad libitum*. Water consumption, food intake and body weight were monitored for any significant changes. Mice were housed in groups (8 animals per group) according to the determinant from the bacteria they were exposed to (e.g., all mice in one compartment would receive the LPS-rich solution only). The two and four week groups were housed within the same compartment with half of the mice removed for each temporal experimental endpoint.

*E. coli* O157:H7 bacteria were grown to OD_600_ 0.2, and then heat-killed. 1.25 ml of bacterial suspension was then added to one litre of water to get approximately 6×10^6^ bacteria/litre. For this study, six treatment groups were created: group 1 received control, tap water; group 2 received heat-killed bacteria; group 3 received DNA prepared from group #2; group 4 received RNA prepared from group #2; group 5 received protein prepared from group #2; group 6 received LPS prepared from group #2. Animals were sacrificed either immediately after treatment (4 animals in each group) or two weeks later (4 animals in each group). The following concentrations were used: DNA at 430 µg/L, RNA at 72.7 µg/L, protein at 9.6 µg/L and LPS at 50 µg/L. DNA extracted from a single *E. coli* cell weighs ∼5×10^−9^ µg, thus 6×10^6^ bacteria would weigh 30×10^−3^ µg, which is ∼15,000-fold less DNA than was used in the experiment. Also, typical bacterial cell contains 0.1 pg of RNA; thus 6×10^6^ bacteria would yield 0.6 µg of RNA, which is 200-fold less than used in our experiment. Average bacterium contains approximately 200×10^−9^ µg of protein [15]; thus 6×10^6^ bacteria would yield 1.2 µg of protein, or 8 times less than used in our experiment. The use of increased concentrations of DNA, RNA and protein was intentional to ensure a large concentration of bacterial components was present in the water to induce a response to the contaminant. Proportionally higher concentration of bacteria in water was not possible to achieve without causing the water to be turbid. The water consumption was comparable among all groups of animals. Consumption of contaminated water did not cause any physiological distress in animals. Animals in the four week test group received normal water for two weeks following initial treatment (Figure S1). Animals were sacrificed either 2 or 4 weeks (depending on the test group) after the start of the treatment. Liver and muscle tissue samples were harvested and processed for molecular testing or fixed in paraformaldehyde for immunohistochemical analysis. The liver was chosen as an indirect target organ, because of its capacity to detoxify the host blood from possible toxins and pathogens [8]. Muscle cells were used as a control that should be neutral to bacterial exposure.

### DNA, RNA and protein extraction

DNA was extracted from the *E. coli* O157:H7 using a Qiagen DNAeasy kit (Qiagen) in accordance with the manufacturer's specifications. RNA was extracted from the *E. coli* O157:H7 using TRIzol® Reagent following the manufactures protocols. For protein extraction, 1 ml of bacterial suspension was centrifuged at 5,000×g for 20 min at 4°C. Next, 500 µl of Lysis buffer (1% Sodium Dodecyl Sulphate) was added and each sample was sonicated for 30 s. Cell debris were removed by centrifugation at 10,000×g for 30 min. Supernatants containing the proteins were transferred to new tubes.

### Lipopolysaccharide extraction

Bacterial cells were harvested by centrifugation (Eppendorf ® 5415R Centrifuge) at the speed of 1,000 rpm for 15 min and LPS was purified as previously described [16]. The procedure for purification of LPS does not completely exclude addition of portions of the bacterial cell wall [16]. Some amounts of other components such as proteins may also be included in the LPS rich solution, therefore the extract is identified as a crude LPS-rich solution.

### mRNA expression analysis and RT-PCR

Total RNA was extracted from 100 mg of the mouse liver tissue using 1 ml TRIzol® Reagent (Invitrogen, Burlington, ON) according to the manufacturer's instructions. Tissue from the four animals per experimental group - exposed for two weeks to LPS, exposed to whole heat-killed bacteria, as well as control animals – were used for the gene expression analysis. The mRNA expression analysis was performed by Genome Quebec (Montreal, QC) with an Illumina MouseWG-6 v2.0 Expression BeadChip. Data produced from the Chip assay was analysed using an Ingenuity IPA Network Analyser and significance was calculated with the use of ANOVA and Significance analysis of microarrays (SAM) test.

RT-PCR was carried out on a Bio-Rad Laboratory's CFX96 Real-Time PCR Detection System (Mississauga, Ontario), using *Taq* DNA polymerase (Fermentas, Burlington, Ontario). Each reaction contained 2 µl of cDNA, prepared with RevertAid^TM^ H Minus First Strand cDNA Synthesis Kit (Fermentas, Burlington, Ontario), 10 pM of forward and reverse primers, 2 mM MgCl2, *Taq* buffer with KCl, and 0.625 units of *Taq* DNA polymerase. Specific primers were designed using integrated DNA Technology primer design software (Oligo Perfect™ Designer) (Table S1). A heat-map showing ANOVA analysis of the mRNA expression, was produced with the assistance of IPA Network® program.

### Immunohistochemical analysis

Paraffin embedding and sectioning of the tissue was conducted at Pantomics (Richmond, CA). Tissue sample labels were recorded and replaced with a random numbered system to ensure no predetermined knowledge was given to either Pantomics or the individual quantifying the data visualized by the fluorescent probes. Upon fixation, the slides were stained with DAPI and immunostained by using either antibodies against phosphorylated γH2AX or antibodies against PCNA (both probes acquired from Santa Cruz Biotechnology, Santa Cruz, CA), as previously described [17].

Specifically, the primary antibody (either PCNA or *γ*H2AX at 1∶500 and 1∶350, respectively) was added to goat serum/1× PBS (1∶200) overnight at 4°C. The slides were washed (similarly to previous cycles) to remove excess antibodies and goat anti-mouse serum (1∶200) for PCNA antibody and anti-rabbit 594 serum (1∶200) for *γ*H2AX antibodies was added.

Samples were examined with a Zeiss confocal microscope and quantified without prior knowledge of the predetermined pattern created by an independent third party. Each tissue sample was digitally sectioned into several equal portions and cells expressing PCNA or *γ*H2AX were recorded by counting. Foci were counted by eye in a blinded fashion by two independent investigators. For *γ*H2AX, at least 100 cells from each sample were examined. The PCNA index was quantified by enumerating PCNA-positive cells in at least 30 high power fields. The data are presented as the fold difference between treated and non-treated cells ± a standard error.

### Western blot analysis

Tissue samples for protein analysis were snap-frozen in liquid nitrogen immediately after animals were sacrificed. Tissues were sectioned (∼25 mg), washed thoroughly, sonicated in 1% SDS and small aliquots of extracts were isolated for protein analysis using Bradford dye reagents from BioRad (Hercules, CA). For western blot analysis, each sample aliquot was standardized to be 2 mg/ml. Western blot analysis was performed as described before [17].

Equal amounts of protein (∼20 µg) were used for SDS polyacrylamide gel electrophoresis at 150 V for 1 h. Smaller predicted proteins such as PCNA (36 kDa) and MeCP2 (53 kDa) were identified using a 12% polyacrylamide gel, whereas KU70 (70 kDa), DNMT3A (85 kDa) and DNMT3B (96 kDa) were identified using a 10% polyacrylamide gel and DNMT1 (138 kDa) with an 8% gel. Specific antibodies used: KU70 and PCNA (both 1∶1000, Santa Cruz Biotechnology, Santa Cruz, CA), POL β, APE1, MeCP2, DNMT1, DNMT3A and DNMT3B (all are 1∶1000, Abcam, Cambridge, MA). Antibody binding was revealed by incubating with horseradish peroxidase-conjugated secondary antibodies (Amersham, Baie d'Urfé, QC) and the ECL Plus immunoblotting detection system (Amersham, Baie d'Urfé, QC). Chemiluminescence was detected by Biomax MR films (Eastman Kodak, New Haven, CT). Unaltered PVDF membranes were stained with Coomassie Blue (BioRad, Hercules, CA), and the intensity of the Mr 50,000 protein band was assessed as a loading control. Signals were quantified using NIH ImageJ 1.63 software and normalized to both actin and the Mr 50,000 protein which gave consistent results. Each protein extract was analyzed three times to ensure significance of the results.

### Analysis of DNA methylation

DNA methylation was analyzed by cytosine extension assay as previously described [18]. The assay utilizes the methylation-sensitive endonuclease *Hpa*II which recognize CCGG sequence and is not able to cut when internal cytosine (at the CpG) is methylated. DNA digested with *Hpa*II leaves a 5′ guanine overhang. Next, the single nucleotide extension reaction with labeled (3H)dCTP fills in the overhang and the degree of (3H)dCTP incorporation is evaluated by measuring radioactive counts. The incorporation of (3H)dCTP inversely correlates with methylation level. In brief, one aliquot of genomic DNA from each liver sample was digested with *Hpa*II, whereas the second aliquot with undigested DNA was used as the background control. The single-nucleotide extension reaction was performed with subsequent measurement of radioactive count as described before [18]. Each reaction for each of 4 animals per single experimental group was repeated twice and the average and SE were calculated.

### Statistical analysis

To identify significant alterations, statistical analysis of the data was conducted for every experiment with a significance confidence level of a minimum of 95% (p≤0.05). A comparison between different treatments was performed, using ANOVA for continuous responses and statistical tests for contingency tables such as Fisher's exact test. The analysis of data was performed using the software packages Stat View and Analyze It for Excel and checked using the statistical analysis program SPSS 15.

## Results

### Exposure to LPS from heat-killed bacteria leads to increased levels of γH2AX

H2AX is a histone variant and its phosphorylated form, γH2AX, serves as an indicator of the DNA strand breaks in the cells [19]. Immunofluorescence analysis of liver cells identified increased levels of γH2AX in animals exposed for two weeks to whole heat-killed bacteria (2.7 fold increase, p<0.05) and LPS (1.95 fold increase, p<0.05) between test groups (Figure 1). Liver cells of animals that consumed tap water for another two weeks (4 weeks group) also exhibited high levels of γH2AX – a 3.25 and 3.3 fold increase was observed in response to whole bacteria and LPS, respectively. Exposure to other bacterial components did not result in an altered level of γH2AX (Table S2). This analysis indicated that liver cells accumulate DNA damage in response to whole heat-killed bacteria or LPS present in drinking water and that the DNA damage continues to accumulate even two weeks after exposure.

**Figure 1:** Immunohistochemical analysis of liver tissue samples stained with DAPI staining and Green Fluorescent antibody for γH2AX. A. Images taken from animals in the group exposed to tap water (control), DNA, RNA, protein, LPS and whole heat-killed bacteria. B. Bars show the average (with SD) fold difference in number of γH2AX-positive cells between treated and control groups. Asterisks show significant difference from control (p<0.05).

### KU70 and APE1 protein levels change in response to whole bacteria and LPS

Elevated level of γH2AX indicates an increase in the level of strand breaks in the liver cells of animals that consumed whole heat-killed bacteria or LPS. To further test whether these additional strand breaks stimulated the increase in amount of DNA repair enzymes, we performed Western blot analysis of KU70, a key protein in the non-homologous end-joining (NJEJ) repair pathway [20]. A 2.5 fold increase was observed upon exposure of the mice for two weeks to whole heat-killed bacteria and a 1.67 fold increase upon LPS exposure (Figure 2A). In contrast, levels of KU70 were not changed in animals exposed to DNA, RNA and protein purified from the heat-killed bacteria. Animals that consumed tap water for two weeks after being exposed to heat killed bacteria or LPS had KU70 levels comparable to the control group (Table S3). These data may be a further indication of the accumulation of the strand breaks in liver cells in response to heat-killed bacteria and LPS.

**Figure 2:** Western blot analysis of KU70 (A), APE1 (B) and PCNA (C) protein levels in liver tissue of mice exposed to whole heat-killed *E. coli* O157:H7 bacteria and DNA, RNA, protein, and LPS extracted from heat-killed bacteria. Bars show the average protein levels (with SD) as compared to the control set at 100%. Asterisks and bars show significant increase from non-exposed controls through the analysis of data using one way ANOVA test (p<0.05). Lower panel shows representative Western blots in 2 and 4 weeks groups.

To test whether exposure to bacteria or its components activates any other repair pathways, we tested the protein level of APE1, involved in base excision repair (BER). A significant decrease in expression of APE1 was identified when animals were exposed to LPS (1.19 fold decrease) and whole heat-killed bacteria (1.13 fold decrease) in the two week group (Figure 2B) as compared to the control. All other components did not result in any significant difference in expression compared to the control (Table S4). In the four week group, levels of expression returned to comparable levels to those seen in the control group (Figure 2B). These data may be an indication that BER activity is suppressed in the liver cells of animals that consumed heat-killed bacteria or LPS.

### Exposure to LPS from heat-killed bacteria leads to increased expression of PCNA in liver cells

Next, we measured the level of PCNA protein. Western blot analysis identified a significant increase in the expression of PCNA in animals exposed for 2 weeks to heat-killed whole bacteria or LPS (p<0.05 in both cases) when compared to the control group (Figure 2C). Analysis of samples from the four weeks group (2 weeks exposure plus 2 weeks normal water) showed that PCNA levels in whole heat-killed bacteria and LPS groups were still increased, as compared to the control, albeit to a lower extent (p<0.05) (Table S5). Other treatment groups did not show any significant alteration in the expression of PCNA.

To support the data obtained by Western Blot analysis, an immunofluorescence analysis of PCNA protein was performed. We also found a substantial increase in PCNA in the liver tissue of animals exposed for 2 weeks to the whole heat-killed bacteria or LPS (Figure 3A). PCNA remained high in the 4 weeks group as well, although the difference was less pronounced as compared to 2 weeks group (Figure 3B, C; Table S6). Exposure to other components of bacterial cell did not result in any change in PCNA levels.

**Figure 3:** Immunohistochemical analysis of liver tissue samples stained with DAPI staining and Green Fluorescent antibody for PCNA. **A**. Images of liver samples taken from individual animals within 2 week and 4 week test groups. B. Quantification of PCNA-positive cells. Bars represent the average (with SD) number of PCNA cells. Asterisks show significant differences from control (p<0.05).

### Exposure to LPS from heat-killed bacteria leads to an increase in expression of maintenance and de novo DNA methylation enzymes and a decrease in global genome DNA methylation

Genome stability in part depends on the degree of chromatin condensation, with the latter depending on changes in DNA methylation and histone modifications. Changes in DNA methylation lead to changes in gene expression as well as in alterations in genome stability.

To analyze the activity of DNA methylation in liver cells, we tested expression level of maintenance methyl transferase (MTase) DNMT1, *de novo* MTases DNMT3A and DNMT3B and protein that binds methylated DNA, MeCP2. Exposure to whole heat-killed bacteria resulted in an increase in the level of DNMT1 protein: 1.71 fold and 1.67 fold increases (p<0.05 in both cases) were observed in the two and four week samples, respectively (Figure 4A, Table S7). Exposure to LPS showed a significant 1.25 fold increase in the two week sample, and a 1.24 fold increase in the four week sample (p<0.05 in both cases). Exposure to DNA, RNA or protein did not change the expression of DNMT1.

**Figure 4:** Western blot analysis of DNMT1 (A), DNMT3A (B), DNMT3B (C) and MeCP2 (D) protein levels in liver tissue of mice exposed to whole heat-killed *E. coli* O157:H7 bacteria and DNA, RNA, protein, and LPS extracted from heat-killed bacteria. Bars show the average protein levels (with SD) as compared to the control set at 100%. Asterisks and bars show significant increase from non-exposed controls through the analysis of data using one way ANOVA test (p<0.05). Lower panel shows representative Western blots in 2 and 4 weeks groups.

The protein level of *de novo* DNA MTase, DNMT3A, also increased upon exposure to whole bacteria and LPS samples. A two week exposure resulted in a 1.96 fold increase for whole bacterial exposure and a 1.25 fold for LPS exposure (p<0.05 in both cases). The analysis of four week samples showed that the levels of DNMT3A dropped and showed no significant alteration for whole heat-killed bacteria and LPS as compared to the control group (Figure 4B, Table S8). All other samples did not have any significant alterations in expression of DNMT3A.

The level of DNMT3B protein, also involved in *de novo* DNA methylation was increased upon exposure to whole bacteria and LPS samples. A two week exposure resulted in a 1.57 and 1.18 fold increase for whole bacterial and LPS exposures, respectively (p<0.05 in both cases). In the four week samples, the expression of DNMT3B increased in response to LPS (1.25 fold, p<0.05) but not to whole heat-killed bacteria (Figure 4C, Table S9). Exposure to other bacterial components did not have any significant alterations in expression of DNMT3B.

Finally, MeCP2 protein levels were significantly increased in response to whole bacteria and LPS. Exposure to the whole heat-killed bacteria resulted MeCP2 expression increased by 1.76 and 1.37 fold in the two and four week samples (p<0.05 in both cases) (Figure 4D, Table S10). LPS levels were also increased in two and four weeks samples –1.2 and 1.28 fold increase was found, respectively (p<0.05 in both cases). All other samples did not have any significant alterations in expression of MeCP2.

To test whether the increase in the expression of methyltransferases would also result in the increase global genome DNA methylation, we performed cytosine extension assay. The analysis showed DNA hypomethylation in the 2 weeks groups exposed to LPS or whole heat killed bacteria (p<0.05 in all cases), but not in the other treatment groups (p>0.05) (Figure S2).

### Exposure to LPS or whole heat-killed bacteria leads to alterations in mRNA expression within liver tissues

Since only exposure to whole bacteria and LPS triggered changes in the expression of genes involved in DNA repair, proliferation and DNA methylation, we performed the microarray analysis only using tissue from animals exposed to whole bacteria, LPS for two weeks and control. As a cut off, we utilized the p<0.05 and fold change of log2>1 (2 fold). Whole heat-killed bacteria exposure increased the expression of interleukin L1, 6, 4, 17B and Tumour Necrosis Factor, and decreased expression of Glycine C-Acetyltransferase genes. LPS exposure increased the expression of *Ccl6*, *Fads2*, *Plin2*, *Pnrc1* and *Rxra* genes. Several transcripts were altered in similar manner upon the exposure to the heat-killed bacteria and LPS. *Dusp1*, *Gadd45g*, *Tff3*, *Esm1*, *Mmd2*, *Gsta1*, *Cyp7a1* and *Alas1* genes changed their transcription levels in response to both whole heat-killed bacteria and LPS (Figure 5).

**Figure 5:** Exposure to LPS and Bacteria alters mRNA levels in mouse livers. A. Clustering of differential expression of genes with the use of control as a standard. Red denotes high expression levels, whereas green denotes low expression levels. RTPCR gene expression analysis of *Dusp1* (B), *Alas1* (C), *Tff3* (D), *Esm1* (E), *Mmd2* (F), *Gsta1* (G), *Cyp7A1* (H), *Gadd45g* (I). Bars show normalized expression levels (average from three reactions, with SD) of aforementioned genes in control and two groups exposed for 2 weeks, whole heat-killed bacteria and LPS groups. Normalization was conducted with Actin transcription levels. Asterisks indicate significant difference (p<0.05).

To confirm the changes in expression of the aforementioned genes, RTPCR analysis was performed. RTPCR confirmed upregulation of the *Dusp1* gene, which was found to be upregulated by 2.7 fold in response to LPS and by 2.2 fold in response to whole bacteria. Results also confirmed an increased expression of the gene *Alas1* in the LPS group but not in the whole bacteria group (Figure 5).

Microarray analysis identified a significant decrease in transcription levels of the *Gadd45g*, *Tff3*, *Esm1*, *Mmd2*, *Gsta1* and *Cyp7a1* genes in both experimental groups. RTPCR analysis confirmed the decrease in the expression in all abovementioned genes, except *Gsta1* expression in the whole bacteria group (Figure 5).

## Discussion

Previously, it was shown that exposure to heat-killed bacteria resulted in an increase in cell proliferation and genome instability of non-exposed liver cells [9]. This research attempted to identify which component of bacteria triggers this response. Exposure to LPS and not to DNA, RNA or proteins resulted in an increase in the level of γH2AX, PCNA, KU70 and DNA methyltransferase proteins. Furthermore, it was identified that a set of 8 genes (*Dusp1*, *Gadd45g*, *Tff3*, *Esm1*, *Mmd2*, *Gsta1*, *Cyp7a1* and *Alas1*) changed their expression upon exposure to whole bacteria and LPS. Below we discuss these findings in details.

### γH2AX, KU70 and PCNA protein levels increase in liver cells of animals exposed to whole bacteria or LPS

Exposure to LPS and heat-killed bacteria caused an increase in the phosphorylation of the H2AX protein. The increase in the γH2AX levels signifies the increase in DNA alteration, mainly DNA strand breaks. Recruitment of γH2AX activates homologous recombination and non-homologous end joining DNA repair pathways [21]. Therefore, it was not surprising to find higher levels of KU70 protein in liver of animals in response to consumption of heat-killed bacteria to parallel higher levels of γH2AX. Our previous research has indicated that pathogenic and non-pathogenic heat-killed bacteria induced higher levels of γH2AX within the liver tissue [9]. Current work demonstrates that a specific component of heat-killed bacteria – LPS – triggers the increase in stand breaks, as reflected by elevated levels of γH2AX and KU70.

It was surprising to see the decrease in the level of BER enzyme APE1 in response to heat-killed bacteria and LPS. Since liver is not an organ that is directly exposed to bacteria or LPS consumed with water (although certain amount of toxins may reach liver cells), it is hard to imagine that bacteria or LPS directly cause the DNA damage in cells. One of many ways the DNA damage may be induced in liver cells is through activation of various signalling molecules, leading to production of radicals and nucleotide oxidation. The fact that APE1 is downregulated in the liver cells in response to bacteria or LPS may suggest that it is unlikely that oxidized nucleotides are formed more frequently in these cells. The downregulation may suggest that there are other types of damages to DNA occur in these liver cells, such as strand breaks, or even that there is no extra damage to DNA. How then one explains the increased level of γH2AX and KU70 in the liver cells of exposed animals? LPS and other endotoxins increase expression of NF-κB that in turn correlates with expression of COX-2 [22]. NF-κB is an inducible transcription factor that regulates a wide variety of genes that have been identified to respond to inflammatory signals [23]. Um *et al*., (2001) has shown that KU70 expression correlates with the expression of NF-κB and COX-2, reflecting high level of cell proliferation [24]. Also, cells with inhibited COX-2 and/or NF-κB genes were identified to have limited ability to repair their DSBs and proliferate [25]. Thus, it is possible that increase levels of γH2AX and KU70 in the liver cells of exposed animals reflect higher levels of DNA replication.

Indeed, the amount of PCNA, a co-factor of replicative polymerase δ, increased in liver tissue after two weeks of exposure to whole bacteria or LPS. It is important to note that PCNA levels remained significantly higher even after two weeks of recovery (four weeks sample). High levels of PCNA may be associated either with an increase in cell proliferation or with an increase in DNA damage. Exposure to LPS can result in direct or indirect damage to DNA via ROS or RNOS pathways [26]. Although we can not rule out the possibility that the increase in PCNA as well as γH2AX and KU70 was due to the increase in the level of DNA damage, the fact that the level of APE1 was not increased, suggests that increased levels of γH2AX, KU70 and PCNA may be due to the increase in cell replication. It is interesting to note that such a response may not necessarily be triggered by direct exposure of liver cells to LPS. In fact, in healthy mice, most of the bacteria and LPS molecules probably do not penetrate the mucous layer of the intestine. It cannot be excluded, however, that a small amount of LPS is absorbed into the portal blood and passed through the liver cells. Healthy intestine is exposed to millions of non-pathogenic *E. coli* cells and thus the host develops antibodies against them; bile and serum in human contain various antibodies against commensal *E. coli* strains [27]. These bacterial strains however do not seem to cause any significant harm, although it should be admitted that studies like the one reported here would be difficult to conduct as mammals are infected with commensal *E. coli* strains in the first hours-days after birth. In contrast, LPS from pathogenic strain does cause serious health problems. For example, LPS has been suggested to be one of the causative agents in inflammation-induced atherosclerosis. Using anti-O157 lipopolysaccharide antibodies, LPS from pathogenic bacteria has been detected in infected humans [28]. Thus, it is possible that the increase in PCNA, γH2AX and KU70 levels is in part due to direct contact of liver cells with LPS.

It is likely that the increase in γH2AX, KU70 and PCNA levels could be due to both, high level of DNA damage and high level of cell proliferation. It should be noted that without continuous exposure to the pathogenic bacteria and/or its components, the levels of DNA damage and thus DNA repair should potentially decrease, requiring fewer proteins such as γH2AX, KU70 and PCNA. In this respect it is curious to note that the levels of γH2AX remained high in animals that received tap water for two weeks after exposure to bacteria or LPS. This may be a further indication that that upregulation of these proteins was largely due to higher cell proliferation activity. Indeed, γH2AX loci are known to form in response to replicative stress – stalled replication fork recruits phosphorylated H2AX [29]. KU70 and PCNA levels decreased in the four weeks group and became similar to control levels.

Exposure to DNA, RNA and protein did not induce any significant alterations in γH2AX, KU70 or PCNA expression, suggesting that these components are unlikely triggering any DNA damage or influencing replication.

### Protein levels of de novo and maintenance methyltransferases increase in liver cells of animals exposed to whole bacteria or LPS

The amount of proteins associated with methylation of the genome, whether due to the *de novo* synthesis (Dnmt3A and Dnmt3B) or maintenance (DNMT1), significantly increased with LPS and bacterial exposure but not in response to other molecules. The constitutive expression of MeCP2 is caused by its ability to perpetuate its own expression. This cycling of expression results in continual expression of the MeCP2 protein and potential to repress genes and manipulate chromatin structure [30]. In this experiment, the expression of DNMT1, DNMT3A and DNMT3B returned to normal levels in animals that were allowed to recover by consuming uncontaminated water for the additional two week period after the initial exposure. This may indicate reversibility of potential changes in DNA methylation. This may also suggest that constant presence of a causative agent, such as LPS, is required for triggering changes in DNA methylation.

The results identify that the naïve cells, distant from the exposed tissue, can be affected by exposure to LPS and whole heat killed bacteria. This indicated that within the two week exposure to multiple components of the bacteria, LPS was identified to be a key bacterial component inducing a response in distal cells and responsible for potential genomic instability. Altered levels of PCNA and γH2AX, increased expression of Ku70 and proteins involved in DNA methylation, in response to bacteria and LPS supported the hypothesis that a bystander-like effect induced genomic instability.

Increase in the expression of MTases could be due to several reasons, including DNA damage and increased DNA replication or/and cell proliferation. Repair of DNA damage as well as replication result in passive loss of DNA methylation that needs to be restored by maintenance DNA MTase DNMT1. Indeed, our analysis showed a decrease in global genome DNA methylation in 2 weeks samples from LPS and whole heat-killed bacteria treatments (Figure S2). Restoration of the methylation levels observed in 4 weeks group is most likely due to the activity of overexpressed methyltransferases. As far as activation of *de novo* DNA methylatransferases goes, it can be suggested that either exposure to bacteria or LPS activate methylation of new CG regions in unreplicated DNA, or these exposures lead to increase in replication that somehow co-regulates the maintenance and *de novo* methyltransferases. In fact, co-culturing of gastric cancer cells with *H. pylori* was shown to activate expression of both, DNMT3a and DNMT1 as well as lead to hypermethylation of tumor suppressor gene WWOX [31]. Another study showed hypermethylation of COX-2 promoter paralleled by DNMT1 overexpression in gastric cancers associated with *H. pylori* infection [32]. Response to viral infection is slightly different. Infection of chickens with Marek's disease virus (MDV) resulted in upregulation of DNMT1, but downregulation of DNMT3B genes [33]. Other papers however showed that viral infection leads to differential regulation of DNMT1, DNMT3a and DNMT3b, with those genes being up- or downregulated, depending on the cell type and the virus type used in the experiments [34], [35].

Exposure to DNA, RNA and protein did not induce any significant alterations in expression of methyltransferases or changes in DNA methylation levels, suggesting that these components are unlikely candidates to trigger changes in epigenetic regulation of response to bacteria.

### Exposure to LPS and whole bacteria result in changes in the expression of eight different genes

Microarray analysis of liver cells in animals exposed to LPS or whole heat-killed bacteria showed differential expression of eight genes that were verified with RTPCR. Altered expression of the eight genes (*Dusp1*, *Gadd45g*, *Tff3*, *Esm1*, *Mmd2*, *Gsta1*, *Cyp7a1* and *Alas1*) could have detrimental effects on the host. *Dual specificity phosphatase 1* (*Dusp1*) expression was found to be altered in fibroblasts exposed to oxidative/heat stress and upon stimulation with growth factors [36]. In this study, Abraham and Clark identified DUSP1 as having a potential role in the cellular response to environmental stress as well as in the negative regulation of proliferation and an inflammatory response. An increase in expression of *Dusp1* may have occurred to assist in the cells' ability to survive the shock of the LPS-induced reaction [37].

An increased expression level of the gene coding for aminolevulinic acid synthase 1 (ALAS1) protein was also identified. This nuclear encoded mitochondrial enzyme is the first and rate-limiting enzyme in the heme biosynthetic pathway (Red Blood Cell (RBC) production). The production of RBCs could accelerate with influx of this specific protein and any other in an eight step process [36]. Tumour cells may increase the expression of enzymes in this process, to assist in the production of RBCs, to oxygenate new tumour cells throughout the body.

*Growth arrest and DNA-damage-inducible 45 gamma* (*Gadd45g*) gene encodes the stress sensor protein that modulates the response of mammalian cells to genotoxic/physiological stress and modulates tumour formation. The transcription of the aforementioned gene is changed in response to stressors inducing growth arrest [38]. GADD45G protein also responds to environmental stresses by mediating the activation of p38/JNK pathway via MTK1/MEKK4 kinase [39]. A decrease in transcription level of *Gadd45g* gene inhibits the production and dimerization of MEKK4, allowing cellular proliferation, differentiation, inflammation and tumourigenesis [40].

Another mRNA with decreased gene transcription level in response to bacteria or LPS was identified as *Tff3* (*Trefoil factor 3*). The function of the encoded protein is not well defined; however it is predicted to stabilize the mucus layer and affect healing of the cells themselves. Recently, TFF3 protein has been identified to be involved in the immune response [41]. This research has identified very low levels of the TFF3 protein during liver and gastrointestinal tissue damage, and high levels of *Tff3* gene transcription briefly after the tissue was repaired. Our analysis showed that the transcription level of *Tff3* was increased within the two week of exposure to whole heat-killed bacteria of LPS. It remains to be shown whether similar changes would be found within the four week sample group.

The expression of the *endothelial cell-specific molecule 1* (*Esm1*) gene coding for ESM1 protein was found to be lower in liver cells from the LPS and whole bacteria group. ESM1 is regulated by cytokines, identifying potential involvement in pathogenic infections. *Esm1* expression has been shown to be increased in the presence of pro-angiogenic growth factors, such as VEGF (vascular endothelial growth factor) or FGF-2 (fibroblast growth factor 2). A significant decrease in transcription of *Esm1* gene, correlates with previously reported decrease in transcription level of pro-angiogenic growth factors such as VEGF or FGF2 genes [42].

*Macrophage differentiation associated 2* (*Mmd2*) gene was reduced in expression for LPS and whole heat-killed bacteria test groups. MMD2 is involved in the immune response and in differentiation of monocytes to macrophages. Since the response to bacteria/LPS may trigger an immediate immune response upon which monocytes differentiate into macrophages, it can be suggested that the expression of *Mmd2* is no longer required at two weeks post exposure. It is possible that *Mmd2* expression was increased in the first two days of exposure and then decreased at two weeks post exposure. It remains to be shown whether *Mmd2* levels would return to normal levels after a two weeks recovery period.

*Glutathione S-transferase alpha 1* (*Gsta1*) mRNA was downregulated in our experiments. GSTA1 has enzymatic functions associated with the detoxification of electrophilic compounds such as carcinogens, environmental toxins and products of oxidative stress. These highly polymorphic enzymes alter the susceptibility of the organism to carcinogens, toxins and alter the effectiveness of some pharmaceutical drugs. The decrease in expression identified in our experiment implicated that the liver tissue was highly susceptible to damage caused by ROS.

Finally, analysis showed a decrease in the steady state RNA levels of the *cytochrome p450 family 7, subfamily a, polypeptide 1* (*CYP7A1*) gene. CYP7A1 is involved in drug metabolism and synthesis of bile acid and steroids from cholesterol within liver tissue. Conversion of cholesterol into bile acid is controlled by this protein and is the main process of removing cholesterol from the body [43]. Removal of cholesterol from the body is important to the overall homeostatic state of organism. Even though there seems to be no connection with an immune response for this particular protein, altered levels may affect the entire organism through inhibition of elimination of cholesterol.

## Conclusion

This work is the first to show that a heat-killed bacterial component known as LPS can lead to distinct molecular changes in the liver. It is important to note, that many changes in liver cells after a two week exposure to LPS returned to levels similar to the control group, indicating the recovery period for such alteration is short. Changes in the levels of protein and expression of mRNAs in liver samples after exposure to whole heat-killed bacteria were more pronounced than after the exposure to LPS. This indicates that LPS may contribute to genome instability caused by bacterial contaminants in the intestine or blood, but it is not the only component. Toxins released by the bacteria upon death may also have some negative effect. Since filtering the water would not remove released toxins (such as Stx1 and Stx2), it is possible that exposure to these toxins may have had an additive effect to changes in the stability of cells in direct contact with the toxins or distal naïve cells. Indeed several reports suggest that Stx1 and especially Stx2 may interact with LPS, thus dramatically increasing LPS toxicity to the cells; injection of mice with the combination of Stx2 and LPS resulted in a severe hemolytic-uremic syndrome (HUS) as compared to a milder effect caused by Stx2 only [43]. On the other hand, injections of LPS only did not lead to HUS and did not cause death in mice, thus suggesting that LPS alone does not cause the renal failure [43]. Since we cannot exclude that the crude LSP extract that we used has a low amount of Shiga toxins, it is possible that the effect of LPS on genome stability and proliferation of liver cells is not purely due to LPS alone but rather due to the potentiation effect of Shiga toxins. The more drastic effect of heat-killed bacteria on liver cells as compared to crude LPS could be due to higher concentrations of Shiga toxins and thus a more drastic potentiation effect between LPS and Stx2.

Another possible product of the bacterial exposure that can impact host cells is circulating inflammatory and anti-inflammatory cytokines produced by affected cells themselves [44]. Further research with the expansion into the inflammatory or anti-inflammatory field is required to identify every component of the bacteria that could induce the effects of carcinogenesis on liver tissue. Another remaining question is whether the bystander effect can induce genomic instability in other organs and tissues throughout the body. Recently, while this paper was accepted for publication, our work demonstrating similar effects of LPS on spleen cells of treated animals was accepted for publication [45]. The study showed that not only liver, but other organs can also exhibit similar response to pathogenic bacterial determinants.

## Supporting Information

Figure S1 **Experimental design to analyze potential genomic alterations induced in the liver cells of mice.** Four-week-old animals received treatment water for two weeks. First set of four animals (per group) was sacrificed immediately after this treatment, whereas the second set of four animals was sacrificed in two weeks, after receiving normal tap water.
(TIF)

Figure S2 **Analysis of global genome DNA methylation.** Global genome DNA methylation was analyzed by cytosine extension assay. The data are shown as the average (from 4 biological and 2 technical repeats with SE) level of incorporation of radioactive dCTP nucleotides (dpm ^3^H). Radioactive counts are inversely proportional to the DNA methylation levels. Asterisks show significant difference between treatment and control groups (p<0.05).
(TIF)

Table S1 **Sequence of the forward and reverse primers for RT-PCR analysis from liver samples.** All primers created with the DNA Technology primer design software (Oligo Perfect™ Designer).
(DOCX)

Table S2 **Imunohistochemical analysis of γH2AX protein expression quantified.** Average±SD represents the average protein expression±standard deviation, compared to the control test detected via analysis of images. Asterisks identify significant increases from non-exposed controls.
(DOCX)

Table S3 **Western blot analysis of Ku70 quantified with Image J. program.** Average±SD represents the average protein expression±standard deviation, compared to the control test. Asterisks identify significant increases from non-exposed controls.
(DOCX)

Table S4 **Western blot analysis of Ape1 quantified with Image J. program.** Average±SD represents the average protein expression±standard deviation, compared to the control test. Asterisks identify significant decreases from non-exposed controls.
(DOCX)

Table S5 **Western blot analysis of PCNA quantified with Image J. program.** Average±SD represents the average protein expression±standard deviation, compared to the control test. Asterisks identify significant increases from non-exposed controls.
(DOCX)

Table S6 **Imunohistochemical analysis of PCNA protein expression quantified.** Average±SD represents the average protein expression±standard deviation, compared to the control test detected via analysis of images. Asterisks identify significant increases from non-exposed controls.
(DOCX)

Table S7 **Western blot analysis of Dnmt1 quantified with Image J. program.** Average±SD represents the average protein expression±standard deviation, compared to the control test. Asterisks identify significant increases from non-exposed controls.
(DOCX)

Table S8 **Western blot analysis of Dnmt3A quantified with Image J. program.** Average±SD represents the average protein expression±standard deviation, compared to the control test. Asterisks identify significant increases from non-exposed controls.
(DOCX)

Table S9 **Western blot analysis of Dnmt3B quantified with Image J. program.** Average±SD represents the average protein expression±standard deviation, compared to the control test. Asterisks identify significant increases from non-exposed controls.
(DOCX)

Table S10 **Western blot analysis of MeCP2 quantified with Image J. program.** Average±SD represents the average protein expression±standard deviation, compared to the control test. Asterisks identify significant increases from non-exposed controls.
(DOCX)
